# Application of Bayesian Algorithm in Risk Quantification for Network Security

**DOI:** 10.1155/2022/7512289

**Published:** 2022-07-08

**Authors:** Lei Wei

**Affiliations:** School of Criminal Justice, Shanghai University of Political Science and Law, Shanghai 201701, China

## Abstract

Network security risk quantification involves both technical and management aspects. Risk quantification has great uncertainty and cannot be fully quantified. Therefore, the fully objective realization of network information security risk quantification is not yet mature. This paper analyzes and quantifies the network security risks caused by various threat sources through a network security risk quantification model based on the Bayesian algorithm. By combining expert knowledge, the conditional probability matrix under the inference rule of the Bayesian algorithm is clarified, and the subjective judgment information of experts on the damage degree of the target information system is synthesized into the prior information system of network security threat. The Bayesian algorithm is used to realize the observation node of objective assessment information and combining subjective security threat levels to achieve continuity and accumulation of security assessments. The error is about 3%, which has a very good effect on the quantification of network security risk.

## 1. Introduction

With the continuous development of network information and the Internet of Things, especially the continuous growth of the Internet information industry in recent years, the quantification of network security risks on the Internet has become more and more important [1, 2]. Problems existing in adopting changes to traditional solutions cannot obtain effective parameters, which leads to the low quantification precision of cybersecurity risk quantification quantitative model, and the optimization of network security risk quantitative parameters is studied by the numerical simulation method. For the host risk calculation, the risk vector is defined according to the state of the host, and a reasonable weight function is obtained through weighted calculation, and the direct risk value and indirect risk value of the host are combined to obtain the host risk value. While communication between different computer networks can increase efficiency, it also presents an opportunity for cyberattacks, a new attack method for systemic security vulnerabilities, widely used by intruders and hackers. In addition, the dangers and threats to information system security are gradually eliminated. Information system security has always been the focus of attention. A large number of intrusions on the Internet make computer users and many organizations face potential network security risks. Therefore, there is a strong need to prevent network systems, organizations, and government agencies from being attacked [3]. An intrusion can be interpreted as an attempt to break into an information system and disrupt various aspects of the system's integrity, availability, confidentiality, or service performance. Organize some preventive measures to protect network systems, servers, and confidential data from intrusion, such as using passwords, firewalls, or strict access control mechanisms to verify the identity of users. These protections are not completely protective because they fail to detect malicious attacks from ill-intentioned workers and cyberattacks, for example, buffer flooding attack, which exploit application feeble and provide great security. The issue of cybersecurity has been a high concern in every country, especially in military needs. The advantage of using a cybersecurity system for evaluation is the wide range of system accuracy postulates. Blurred set theory and blurred logic have become effective methods for quantitatively representing and dealing with inaccurate choices. A blurred set or blurred number can properly represent inexact parameters and can be manipulated by various operations on the fuzzy set or fuzzy number. The comprehensive assessment mode of computer network communication security is a matter of collective efforts. Group decision-making (i.e., multiple experts) is typical decision-making behavior. Using this expert can alleviate some decision-making difficulties caused by complex and uncertain problems [4–6]. Group decision-making problems tend to follow a general solution consisting of two phases: the aggregation phase and the development phase. Many aggregation operators and methods have been developed to solve group decision problems with linguistic information. It can effectively avoid information loss and false positives in the process of language information processing. The Bayesian algorithm embodies the simple statement of conditional independence that each variable is an autonomous nondescendant in the graph given its parent state. This feature can be used to reduce (sometimes greatly) the number of various parameters required to characterize a variable. Such an algorithm provides an efficient way to calculate the posterior probability. Effective decision-making and quantitative assessment of network information security risks are one of the effective ways to solve security problems in information systems. Information security assessment is the application of risk assessment theory and method in the information system. Including fault tree analysis, AHP (analytic hierarchy process), and fuzzy comprehensive evaluation, information security assessments have been used by reviewers. Through the assessment, let the masses discover the problems and contradictions in information security, and the methods and measures to solve these problems. Therefore, the information security evaluation is very important to improve the security significance of the information system. However, to date, the impact of human factors and management measures in the area of information systems have not been fully considered. Meanwhile, information security threat assessment involves both technical and management aspects. The assessment is subject to significant uncertainty and cannot be fully quantified. As such, it is difficult to achieve a fully objective cybersecurity risk assessment. This research integrates subjective and objective cybersecurity assessment messages and establishes a quantitative model of network security threat assessment based on the Bayesian algorithm. First, the decision-making method fully draws on the experience and evaluation by every decision maker to evaluate the target intelligence system, which largely makes up for the singularity of the decision-maker's individual judgment; second, compared with neural network, Bayesian network (BN) can completely describe human reasoning process. Dynamically reflect the risk of the system, and if the attack firewall is blocked by the firewall, it will not affect the internal network. Even if the internal network is imperfect, there is no risk under the protection of the external firewall, which ensures the security of the network to the greatest extent. For different network settings of different matrix parameters, different risk assessment results will be obtained after setting the state transition matrix, observation matrix, and initial state, which can adapt to different network environments and is universal. The calculation amount of the model is very small, and the calculation process can be completed in a very short time, which ensures the real-time assessment and real-time reflection of network risk. However, it is difficult to control the size of the observation matrix and associate the observation matrix with the state transition matrix. The safety evaluation based on the Bayesian algorithm can not only explain the safety evaluation process quantitatively, but also embody the accumulation and continuity of safety evaluation [7–9]. Therefore, the information security quantitative model based on the Bayesian algorithm can fully taking into account the subjective judgment data of various decision makers, and it can also prove the continuity and accumulation of safety assessment. In addition, the confidence of the prior information of the Bayesian algorithm is improved.

## 2. Network Security Risk Quantification

In recent years, with the rapid development of electronic communication technology and networks, the national security boundary is not limited to geographic space, but extends to information networks. The network is becoming an increasing number of important in people's lives, and the issue of network security issues cannot be ignored. Nowadays, the network system needs to ensuring the security of network communication, and first of all, it is necessary to make a correct assessment of the network risk. In order to quantify the network risk value and evaluate the threats in the process of network operation, optimizing real-time cybersecurity risk quantification methods were invented. In the past, it was set manually, and now the new method is to set the parameter matrix. The set parameter matrix simplifies the complexity of the configuration. Network security has become an important issue closely related to national security. Therefore, how to accurately quantify the security risks existing in the network, take defensive measures accordingly, as shown in Figure 1, and minimize the losses caused by network security risks as much as possible have become the key issue of relevant scholars' research, and its research has a high degree of importance value. Generally speaking, the measurement of network security risks was achieved through establishing a model. It was impossible to obtain reasonable and effective important factors, and the result of measurement was not reliable. In view of the disadvantages of the traditional methods, some of them introduced the artificial intelligence into the study of network security risks, mainly including the methods of the artificial nerve network and the methods of the support machine. The artificial neural network method has a good approximation ability to nonlinear functions. It is realized on the basis of assuming that the empirical risk is minimized [10–12]. However, the risk cannot be minimized. It has certain defects in theory, which is not good for the quantitative results. It will also cause a certain delay. The support vector machine method is better than the artificial neural network method in solving this kind of problem and has a good expansion ability, but its parameters are relatively large, and the problem can be solved by optimizing the parameters. In view of this, according to the characteristics of the nonlinear characteristics of network security risk, the delay parameter is introduced, and the important parameters of the support vector machine model are optimized through numerical simulation, so as to improve the quantization accuracy. The experimental test is used to verify the performance of the network security risk quantification model after parameter optimization on the actual network security risk quantification.

Based on the Bayesian model, the quantification and optimization of the network security risk assessment method are realized, and based on the Bayesian model, the network security risk quantification method is described in real time, the shortcomings are analyzed, and optimization measures are proposed. The innovation and practicability of this method are presented. It is proved that the risk description rule base can get the optimal solution and can be well used for risk assessment. The research roadmap of this paper is shown in Figure 2. Bayes' rule offers a way to calculate the hypothesis probability with the priori probability. The best assumption is the most likely hypothesis because there are prior probabilities for various hypotheses *h* on the data *D* to be observed, and *h* is the hypothesis space that contains the objective function. The Bayesian algorithm (BA) has many probability classes method and an optimal method for predicting the class of unknown samples [13–15], widely used in data deep search, image processing, bioinformatics and multitarget retrieval of information, and other fields. Look at how the conditions are collected in the data set, and find out which data belong to the different categories using how the conditions are collected. Based on a comprehensive analysis of current research challenges, this time a new algorithm was adopted that uses the Bayesian algorithm to solve problems such as classification rate and false positive rate [16, 17]. Bayesian networks (BN) are used to represent dependencies between nodes using Bayesian theory, which can be represented by variables. BN consists of nodes, arcs, and a node probability table (NPT). Arcs represent causal relationships, and NPTs represent probability tables that summarize the probabilities of occurrence between causal nodes [18, 19]. BN is very useful for solving problems such as insufficient information, a posteriori inference, and the change from qualitative to quantitative problems by learning new knowledge about the relationship between posterior and prior probabilities.

Bayesian networks (BN), also known as directed acyclic graph models (or simply Bayesian network), consist of a series of combinations that express causal rules, and BN corresponds to another GM structure called Directed Acyclic Graph (DAG), belonging to the model series of probability graphics [20–22]. This structure is very popular in statistics, machine learning, artificial intelligence, etc. Bayesian networks can efficiently represent and compute a joint probability distribution (JPD) over a set of random variables. These structures were used to express the places with relative uncertainty. From the picture, it could be seen that each node represented a random variable, and the boundaries between the probability of each node corresponded to the random variable were relevant. The conditions in the picture depended on the estimation, and they usually used the known statistics and calculation techniques. Therefore, Bayesian theory combines principles such as graph theory, probability theory, computer science, and statistics, and GMs with undirected edges are often referred to as Markov random fields or Markov networks. These networks are based on the concept of Markov chains, which provide a simple definition of independence, that is, between any two different nodes [23–26]. The formulas for calculating the mean relative error MAPE and the root mean square error RMSE are as follows:

(1) $$\begin{array}{c} \text{MAPE}=\frac{1}{n}\sum_{i=1}^{n}\frac{\left|y_{\text{true}}^{\prime }-y_{\text{estimate}}\right|}{y_{\text{true}}}\times 100\%,\\ \text{RMSE}=\sqrt{\frac{1}{n}\sum_{i=1}^{n}{\left(y_{\text{true}}^{\prime }-y_{\text{estimate}}\right)}^{2}}, \end{array}$$

where *n* is the total number of samples, *y*_true_′ is the true value, and *y*_estimate_ is the estimated value.

The set *u* is the mathematical expectation assigned to the weight vector *ω* = (1/*n*, 1/*n*,…, 1/*n*, 1/*n*), *σ* is the standard deviation between *u* and *ω*, and there are

(2) $$\begin{array}{c} u_{n}=\frac{1}{n}\frac{n\left(n+1\right)}{2}=\frac{n+1}{2},\\ \sigma_{n}=\sqrt{\frac{1}{n}\sum_{i=1}^{n}{\left(i-u_{n}\right)}^{2}},\\ \omega_{n}^{\prime }=\frac{1}{\sqrt{2\pi \sigma_{n}}}e^{{\left(i-u_{n}\right)}^{2}/2\sigma \pi },\\ \omega =\frac{\omega^{\prime }}{\sum_{i=1}^{n}\omega^{\prime }}. \end{array}$$

In the above formula, *u*_*n*_ is the mathematical expectation, *σ*_*n*_ is the standard deviation, *ω*_*n*_′ is the distribution function, and *ω* is the importance quantification value.

## 3. Analysis of Bayesian Model Results

Network security means that the hardware or software of the network and the data in its system are protected from property loss and personal safety due to accidental or malicious damage, so as to maintain the continuous and reliable operation of the system. Network security should include enterprise (company) security system, transmission security, data security, firewall security, server security, etc. If you want to realize that the personal information (such as bank account number and ID card information) or login information transmitted on the network will not be found by others, you must ensure that the system software, application software, and database have certain self-protection functions, and ensure that these applications cannot be accessed without authorization. In the real world, there is no absolute network security. Especially, in the case of developed network technology, it is a major issue that must be carefully considered to prevent all forms of hacker attack. Everyone has the same definition of network security, but from different perspectives. For enterprises, if there are network security problems, it may cause heavy losses to enterprises; for the country, it may damage national security. To solve these network security problems, programmers need to make great breakthroughs in technology and improve and deal with all kinds of sudden software security problems in time.

The characteristics of the new network security risk are as follows: all kinds of homogeneous and heterogeneous data are widely collected, stored, analyzed, and applied, and data have increasingly become an important strategic resource and new production factor. Information systems and platforms show the characteristics of huge data storage scale, diverse data types, fast data generation speed, and high data value. These valuable data will become the target of criminals' crimes, and the problem of data security will become more prominent in the era of big data. In the context of the Internet and cloud platforms, information virtualization not only promotes the development of the “four new economies” but also makes network security risks more hidden. For example, online pyramid schemes, online drug trafficking, virtual currency, and ransomware based on the Internet platform are characterized by strong concealment, fast transmission speed, virtualization, difficulty in obtaining evidence, a wide range of cases involved, and strong anonymity. The Internet, industrial Internet, and Internet of Things have become “new infrastructure.” The network environment under the new infrastructure is becoming more and more complex and heterogeneous. Although personalized services can be provided according to users and business needs, with the increasing of various network attack means, the need for security is increasing in all key links of heterogeneous networks. The innovation of artificial intelligence technology promotes the development of “four new economies,” and interweaves the traditional network security risks with the new network security risks. The relationship diagram is shown in Figure 3. Information and intelligent technology are a double-edged sword, which not only brings new network security risks, leads to the increase of new intelligent network attack means, but also promotes the formation of new network security governance means.

Different from traditional risks, network security risks are systematic and interdependent and have both high-frequency low-loss and low-frequency large losses. However, traditional risk assessment methods can still be used for reference, and network security risks have been preliminarily described. The probability of reaching the final result gives several relevant evidence variables. The final result possibly encoded into the model along with the probability of occurrence of the evidence variable [27–29]. Assuming that the final result is generated, the probability of the evidence variable is independent of the probability of other evidence variables giving the final result, and the decision-making group is composed of four experts, and the evaluation target is the highest TL [30, 31]. Assuming that the target TL is high, medium, and low, the quantitative judgment information provided by the four decision makers is as follows:

(3) $$\begin{array}{c} U_{1}=\left(0.3,0.5,0.3\right),\\ U_{2}=\left(0.2,0.5,0.3\right),\\ U_{3}=\left(0.37,0.2,0.3\right),\\ U_{4}=\left(0.3,0.6,0.33\right). \end{array}$$

In the formula, *U*_1_, *U*_2_, *U*_3_, *U*_4_ represent the matrix value under different attack strategies. According to the equation, the operator weight vector *w* can be obtained:

(4) $$\begin{array}{c} w=\left(0.123,0.367,0.432\right). \end{array}$$

Among them, *w* is the arithmetic weight operator.

Then, the TL evaluation value *U* of the decision-making group is

(5) $$\begin{array}{c} U=\left(0.245,0.356,0.352\right). \end{array}$$

In the formula, *U* represents the combined attack value.

As shown in Figure 4, the state collection of the variables in the model looks as follows:

(6) $$\begin{array}{c} \text{TL}=\left\{\text{High},\text{Medium},\text{Low}\right\},\\ C=\left\{\text{Big},\text{Middle},\text{Small}\right\},\\ T=\left\{\text{High},\text{Midium},\text{Low}\right\}. \end{array}$$

In the above formula, the threat level is TL, and *C* and *T* are state variables.

The average risk value of the entire network at time *t* is

(7) $$\begin{array}{c} \bar{R\left(t,j\right)}=\frac{1}{L}\sum_{l=1}^{L}R_{l}\left(t,j\right),\;1\leq j\leq 10. \end{array}$$

The host risk value is recorded as *R*_*l*_(*t*, *j*), *L* is the number of units, and $\bar{R_{l}\left(t,j\right)}\;$ is the average host risk.

The risk-independent situation is the same. In the risk-dependent situation, with the increase of the confidence level, the VaR value and ES value of network security incident losses gradually increase. When the confidence level is low, as shown in Figure 5, the splice distribution and the mixed distribution have smaller basic VaR and ES values in describing the loss of network security events, so they are better than the thick-tailed distribution in describing the loss of network security events. When the confidence level is high, the splicing distribution and the thick-tailed distribution are basically the same in describing the loss of network security risk; that is, the VaR value and the ES value are in the same order of magnitude, while the mixed distribution has a smaller VaR value. Therefore, under the condition of network risk dependence, when the confidence was high, the mixed distribution could better describe the loss risk of network security events.

Network security incidents originate from threats and vulnerabilities. The possibility of incidents can be determined by evaluating threats and vulnerabilities of information via algorithms. At the same time, the impact of network information protection incidents is related to funding, and conclusions can be drawn through funding assessment. As shown in Figure 6, information security risk can be regarded as the impact on capital. To simplify the model, only the following factors are considered: impact on capital, frequency of threats to capital, vulnerability of capital F, and threat level TL. In this case, a quantitative evaluation model of information security based on the Bayesian algorithm is established.

There are many hosts in a network. Due to the different importance of the location, the services provided, and the importance of storing and processing data, the importance of the hosts must be different. If an ordinary host at the edge of the network is attacked or completely damaged, there should be no significant impact on the risk status of the network [32]. The impact of network risk was also great. Therefore, in order to figure out the different impact of different host on the network risk and more accurately describe the network risk, the relative importance of the host was introduced, and the traditional calculation method of network risk was modified and weighted. In this way, the risk changes of the entire network can be reflected more realistically, and focused remedial measures can be taken to improve the efficiency of developing security policies.

Analysis of Figure 7 shows that, compared with the comparative literature methods and methods, the method in this paper is most consistent with the quantification value and time results of network security risk, and there are only few differences, while the risk quantification results of different methods and the actual results are very different. The main reason is that the parameters optimized by the method in this paper are the most reasonable, which can make the quantitative results tend to the actual values. Through a more objective analysis of the reliability of the method in the network security risk quantification results, the optimization performance of the method in this paper for important parameters is verified.

The spliced distribution is more sensitive to the change of the shape parameter. When the shape parameter becomes larger, its mean, variance, VaR, and ES values increase exponentially, while the results of the thick-tailed distribution and the mixed distribution are relatively stable, like Figure 8. For thick-tailed distribution, when the shape parameter increases, its mean, variance, VaR, and ES values increase; for mixed distribution, when the shape parameter increases, its mean, variance, VaR, and ES values change slightly mildly, so the mixed distribution has good robustness in parameter setting.  Figure 9 compares and analyzes the probability distribution of network security risk losses under risk dependence and risk independence.

Figure 10 shows that under risk independence, the splicing distribution can better reflect the possibility of the extreme importance of the network security event, but the extreme importance of the splicing distribution is still lower than the possible extreme value of the mixed distribution. Figure shows that, under the risk dependence, both the spliced distribution and the mixed distribution show good thick-tailed and extreme value characteristics. Based on the average risk value at a certain moment, a qualitative model of network security was established by using the support machine with time delay. Then, the important factors in the model were optimal with the combination of the ant group method and the simulation method. The test results show that the method has excellent parameter optimization performance and high network security risk quantification accuracy.

Compared with the change of network risk, the change of risk value calculated by the traditional method is relatively gentle, like Figure 11. The disadvantage of this quantitative method is that network administrators will only notice that it is too late to adopt remedial strategies when the network risk value exceeds the alert value. As shown in Figure 12, the average risk value of the network calculated by the method in this paper varies greatly from time to time. The reason is that the absolute value of the risk of relatively important hosts in the network does not change much, but because of its high weight, it can be caused by the new calculation method. Therefore, the advantage of the method in this paper is that it can detect significant changes in network risks as early as possible, highlight the impact of important hosts on network risks, and achieve focused protection, which is of great significance for improving the security of the entire network and adopting corresponding security strategies in a timely manner.

Most of the existing network security risk measures are qualitative analysis or single loss distribution representation, but this way of thinking ignores the characteristics of system city, interdependence, and network security risk with both high-frequency and low-frequency losses and low-frequency huge losses. Based on the Bayesian method, this paper quantitatively evaluates the network security risk loss. The research results show that the network security risk loss has thick tail characteristics, and the splicing distribution can better describe the extreme events of the network security risk than the single distribution; and the mixed distribution is better than the splicing. Distribution is more advantageous in risk assessment and safety capital preparation. In the case of independent risk, the spliced distribution can better estimate the loss of network security risk; while in the case of dependent risks, the mixed distribution can better describe the loss of network security risk. In addition, the parameter sensitivity analysis of the distribution shape shows that the mixed distribution has good stability, and the distribution can better describe the extreme value and thick-tailed characteristics of network security risk loss. The Bayesian model is an effective method to quantitatively analyze network security risk losses, and its results can guide enterprises to conduct corresponding network security risk management.

## 4. Conclusion

Cybersecurity risk quantification is the basis and premise of network system security management. Aiming at the problem of ignoring the correlation and difference of nodes in traditional quantitative assessment methods, a node-related network security risk quantification method is proposed. In this method, the network node correlation is introduced into the quantitative assessment process based on the hidden Markov model, which solves the problem that the node correlation is generally ignored in the existing quantitative assessment methods of network security risk, characterizes the differences in the contribution of different hosts to network risk. The early network security risk quantification model did not take into account the relatively personal threat evaluation information given by decision makers in professional experience. This is a loss of information for the overall evaluation model. Based on the systematic analysis of information security threat factors, this model combines subjective TL judgment information and objective situation information to establish a network information security risk quantification model based on Bayesian operator. The actual process of information security risk quantification can more accurately reflect the real TL. Bayesian network has been widely used in the field of prediction evaluation. Many scholars use the Bayesian network to conduct network security prediction evaluation research, and gradually become practical. However, the Bayesian network still has the following problems to be solved when it is used in the field of prediction evaluation: (1) in reality, the Internet is constantly changing, but the standard Bayesian network is a static model. Therefore, how to make the standard Bayesian network predict dynamic network security is a worthy research direction. (2) In the study of Bayesian network knowledge synthesis, we maintain the network structure unchanged; that is, we assume that the network structure can describe the problem domain well. However, when the uncertainty knowledge is not consistent with the network structure and comes from unreliable data sources, it may not reflect the problem model realistically. How to combine the related algorithms of Bayesian network structure and realize the synthesis of uncertainty knowledge by modifying the network structure is also a very meaningful research direction. (3) In Bayesian network prediction, efforts are still needed to encode expert knowledge. That is, the Bayesian network needs to be solved. On the one hand, it overcomes the static limitations of the expert system, and it is better to realize knowledge storage, acquisition, and update. The new and more reliable probability knowledge updates the existing Bayesian network and enhances the practical significance of the Bayesian network. The method of quantifying network security risk in real-time provides an effective method for network administrators to manage the network. You can monitor the status of the network at any time, discover network risks, and solve them in time. This paper makes some optimizations and improvements on the basis of the Bayesian method, which makes this method simpler to use and more reliable in parameter setting and evaluation. In the research, it is found that the algorithm of threat degree can classify the types of attacks, and by sorting the degree of threat, the attention of the network maintenance system to irrelevant attacks can also be reduced. The threat algorithm is subject to further modification and testing. With the rapid development of the network, the speed of maintaining network security cannot keep up with the speed of network development. In the future research, it is necessary to reduce network risk, strengthen the research of network risk identification and self-healing, realize the automation of network system maintenance, and meet the needs of most network users. Combined with the relevant algorithms of Bayesian network structure, the uncertainty in network security quantification is realized by modifying the network structure.

## Figures and Tables

**Figure 1:** Study network system structure.

**Figure 2:** Discussion on the research roadmap.

**Figure 3:** Risk quantification diagram.

**Figure 4:** State collection diagram of variables in the model.

**Figure 5:** VaR values in different states.

**Figure 6:** Unequal variance curve.

**Figure 7:** Quantitative value of network security risk.

**Figure 8:** RMSE values under different parameters.

**Figure 9:** Different parameter values under risk independence.

**Figure 10:** Random number of network attacks.

**Figure 11:** Network random frequency statistics.

**Figure 12:** Statistics of network security risk value.

## Data Availability

The data used to support the findings of this study are available from the corresponding author upon request.
